This article has been retracted.

# Acupuncture Combined with Traditional Chinese Medicine and Drug Therapy for the Treatment of Cerebral Infarction (Phlegm-Blood Stasis Syndrome) and Carotid Atherosclerotic Plaque: A Preliminary Randomized Controlled Study

**DOI:** 10.1155/2022/5143408

**Published:** 2022-06-15

**Authors:** Wentong Wang, Zhuli Liu, Yongxiong Wu

**Affiliations:** ^1^Department of Encephalopathy, Shenzhen Hospital, Beijing University of Chinese Medicine, Shenzhen, Guangdong 518100, China; ^2^Inpatient Dispensary, Wuyi Traditional Chinese Medicine Hospital, No. 30 East Huayuan Road, Jiangmen, Guangdong 529000, China

## Abstract

Carotid atherosclerotic plaque (CAP) is one of the leading causes of cerebral infarction. Western medicine usually uses lipid-lowering drugs to stabilize plaques. Currently, studies reporting on drugs that can reduce plaques are lacking. Here, we performed a randomized controlled study to investigate the effectiveness of acupuncture combined with drug therapy (TCM and Western) to treat cerebral infarction (phlegm-blood stasis syndrome) and CAP. The control group was treated with atorvastatin calcium tablets (20 mg/d, po for 15 days). The treatment group received atorvastatin calcium tablets 20 mg, traditional Chinese medicine (TCM) decoctions (two matured substance decoction plus peach kernel and Carthamus four substance decoction plus Chinese hawthorn fruit 20 g, gold theragran 20 g, and red yeast rice 3 g), and acupuncture therapy, once daily for 15 days as one treatment course. The patients' neurological deficit score, ultrasonic testing of the carotid artery, and lipoprotein-associated phospholipase A2 (Lp-PLA2) were evaluated. Our findings showed no significant difference in the evaluated indices between the two groups before treatment (*P* > 0.05). However, compared with the control group after 15 days of treatment and within each group before and after treatment, the differences were significant (*P* < 0.05). In conclusion, acupuncture combined with drug therapy demonstrated promising effectiveness in treating cerebral infarction (phlegm-blood stasis syndrome) and CAP.

## 1. Introduction

Cerebral infarction (CI), also known as ischemic stroke, has been reported to rise at an annual rate of 8.7% in China [1]. However, economic development and measures such as improved blood pressure control, smoking ban campaigns, and widespread use of statins have significantly reduced the risk of fatality from 1984 to 2004 [1–3]. Atherosclerosis is a significant cause of IC. Some studies have demonstrated that hemodynamic changes caused by the formation of carotid atherosclerotic plaque (CAP) are closely related to CI [4, 5].

Traditional Chinese medicine (TCM) has been used in traditional Chinese clinical practice [6]. The basis of TCM is an individualized treatment based on syndrome differentiation by examining the patient's symptoms, investigating the pathogenesis, and determining the disease characteristics and location [7]. Theories of meridians, organs, and stages are employed to differentiate symptoms [8]. In general terms, TCM treatment can be defined as the process of weighing the cons and pros of a patient condition and correlating them with therapeutic principles for individualized Chinese herb prescriptions via oral herbal medicines and nutrition or methods using moxibustion, acupuncture, acupressure, etc. Based on the guidelines from experts of the Chinese Society of TCM, it can treat 95 major diseases, including high incident diseases related to angiogenesis, such as ischemic diseases and diabetic ulcers [9, 10]. Thus, TCM formulas, extracts, and compounds, till present, have a great contribution to the Chinese health to fight diseases in modern society.

Lipids and lipogenesis have been associated with several ailments [11–14]. Western medicine uses lipid-lowering drugs to stabilize plaques, but removing the plaques has shown controversial results as the drugs used may have a short half-life and significant adverse events [15–17]. In TCM theory, CI is classified as “stroke,” with the common symptom being blood stasis, and thus, drugs promoting blood circulation are used to remove blood stasis; lowering lipid levels, soothing the liver, and regulating Qi are used to treat CI [18, 19].

In our clinical practice, we observed that cases with CAP could be cured using TCM therapy, but currently, there is no report of CAP resolution using TCM in the literature. Thus, in this study, we performed acupuncture combined with drug therapy for the treatment of CI (phlegm-blood stasis syndrome) and CAP. Further, as numerous studies have reported that lipoprotein-associated phospholipase A2 (Lp-PLA2) is involved in the formation, progression, and rupture of atheromatous plaque [20–24], this marker was objectively used to evaluate its efficacy of treatment and CAP status.

## 2. Materials and Methods

### 2.1. Patients and Clinical Data

Outpatients and inpatients treated from January 2016 to January 2019 at the Shenzhen Hospital of Beijing University of Chinese Medicine (Shenzhen, China) were assessed. A total of 60 patients with CI (phlegm-blood stasis syndrome) were enrolled in this preliminary randomized controlled trial, and informed consent was obtained from all patients.

The study flow chart is shown in Figure 1. The inclusion criteria were as follows: (1) clinical diagnosis of acute-stage CI based on the criteria of the *Internal Medicine* [25] and confirmed by head radiology at the hospital; (2) fulfilled the diagnostic criteria of phlegm-blood stasis syndrome according to the *Standards of Diagnosis and Therapeutic Effect for Diseases and Patterns in Chinese Medicine* developed by the National Administration of Traditional Chinese Medicine in 1994; (3) underwent carotid ultrasonography which confirmed the presence of CAP (i.e., soft, heterogeneous mixed, and flat plaques); (4) were aged between 40 and 80 years old; and (5) provided written informed consent for the study. The study exclusion criteria were as follows: (1) the onset time was >2 weeks; (2) the patients had a history of severe liver and renal diseases; and (3) the patients were unconscious or unable to cooperate with the study protocols.

### 2.2. Treatment Methods

The patients were randomly and single-blindly assigned to a control or treatment group. The course of the disease was within 2 weeks. Both groups received conventional treatments, including general treatments such as oxygen therapy, lowering intracranial pressure; controlling blood pressure, glucose, and lipid medications; and maintaining water-electrolyte balance, symptomatic and supportive treatments, and 100 mg of aspirin enteric-coated tablets (po, qd).

The therapeutic regimen for the control group included atorvastatin calcium tablets (Pfizer Pharmaceuticals Co., Ltd., NMPA approval number: H20051408), which was orally administrated at 20 mg/d.

The therapeutic regimen for the treatment group was as follows: (1) similar to the control group, the patients were given atorvastatin calcium tablets which was orally administrated at 20 mg/d, and (2) other treatments were as follows: oral TCM decoctions, including Two Matured Substances Decoction plus Peach Kernel and Carthamus Four Substances Decoction plus or minus; prepared using 10 g of pinellia tuber, 20 g of aged tangerine peel, 20 g of poria, 10 g of peach kernel, 5 g of safflower, prepared 20 g of rehmannia root, 10 g of red peony root, 15 g of Sichuan lovage root, 10 g of Chinese angelica, 20 g of Chinese hawthorn fruit, 20 g of gold theragran, 3 g of red yeast rice, 5 g of licorice root. The decoction method included (1) decoction with 200 mL warm water and 100 mL/time, twice a day; (2) acupuncture at the Zúsānlĭ (Zusanli, ST 36), Fēnglong (Fenglong point, ST 40), Hégŭ (Hegu point, LI 4), and Nèiguān (Neiguan point, PC 6). The treatment was performed once a day, 30 min each time, and 15 times repetition was considered as one treatment cycle. The treatment course in both groups was 15 days.

### 2.3. Outcome Measures and Methods

The main outcome was the intima-media thickness (IMT) of the bilateral common carotid arteries, which was measured three times during follow-up using carotid ultrasonography. The average value was utilized for analysis. The secondary outcomes included the following: (1) clinical efficacy: the National Institutes of Health Stroke Scale (NIHSS) and neurological deficit score were used to evaluate the efficacy; (2) value of Lp-PLA2; and (3) safety indices (the three main routine examinations included electrocardiogram (ECG), liver, and renal function tests). The above indexes were recorded and collected once on days 1 and 15 of inclusion.

### 2.4. Statistical Analysis

Measurement data were presented as mean ± standard deviation ($\bar{x}\pm s$) and compared by the paired *t*-test; *c*^2^ test was used for the comparison of enumeration data. Ridit analysis was used for ranked data. Statistical analyses were performed using the SPSS 20.0 software (IBM Co.).

## 3. Results

### 3.1. Study Population and Clinical Characteristics

Sixty patients were randomly and single-blindly assigned to a control or treatment group. The study comprised 30 males and 30 females, and there were 30 cases in each group. The mean age of the patients in the treatment and control group was 54.67 ± 9.736 years and 54.20 ± 8.54 years, respectively.  Table 1 illustrates the basic information between the two groups. No significant differences were detected in the gender, age, course of the disease, and other general data between the two groups (*P* > 0.05; Table 1). All patients were followed up for 2 weeks after the treatment.

### 3.2. Treatment and Outcomes

#### 3.2.1. Flowchart of Participants

There were no dropouts before and after treatment in the two groups of this study.

#### 3.2.2. IMT of CAP

The IMT was the primary outcome and was measured via carotid ultrasonography. The assessment was performed thrice during follow-up, and the average value was utilized for analysis. Our results showed that at 15 days after treatment, the IMT of CAP in the two groups was significantly lower than before treatment (*P* < 0.001). In the treatment group, the CAP was significantly lower than that of the control group over the same period (*P* < 0.001, Table 2).

#### 3.2.3. Lp-PLA2 Value

As Lp-PLA2 has been shown to be a promising marker to evaluate the efficacy of treatment and CAP status, it was employed in this study. At 15 days after treatment, our findings showed that the Lp-PLA2 value in the two groups was significantly lower than before treatment (*P* < 0.001). Further, in the treatment group, the Lp-PLA2 value was significantly lower than that of the control group during the same period (*P* < 0.001, Table 3).

#### 3.2.4. NIHSS

In this study, the NIHSS was employed to assess the clinical efficacy of the procedures performed between the treatment and control groups. At 15 days after treatment, our findings showed that the NIHSS in the two groups was significantly lower than before treatment (*P* < 0.001). Additionally, in the treatment group, the NIHSS was significantly lower than the control group over the same period (*P* < 0.001, Table 4).

#### 3.2.5. Safety Indexes and Adverse Reactions

The results of the three main routine examinations, i.e., ECG, liver, and renal function tests, were unremarkable between the two groups. No adverse reactions, such as rhabdomyolysis, occurred in any of the treatment groups.

## 4. Discussion

In this randomized controlled trial, our findings suggested that acupuncture combined with drug therapy for the treatment of CI (phlegm-blood stasis syndrome) seemed to be more effective compared to single Western medicine drug in alleviating the clinical symptoms, reducing CAP volume, decreasing Lp-PLA2 value, and reducing the risk factors associated with CI recurrence.

Previous studies have focused mainly on the effects of lipid-lowering drugs in CAP and blood lipid analysis, and only a few reports are available regarding TCM therapy [26–28]. Thus, in this study, we used acupuncture, TCM, and Western medicine to investigate the potential efficacies of TCM drugs and methods, compared to Western drug only, and in relation to CAP. The characteristics of CAP in CI patients are related to TCM phlegm-blood stasis syndrome [29]. Phlegm syndrome has been shown to be associated with various diseases, and blood stasis can occur after a long time; thus, CAP belongs to the category of “phlegm-blood stasis” of TCM [30, 31]. The following treatments implemented in this study showed promising results in resolving phlegm and reducing stasis: two matured substance decoction for reducing phlegm-damp, peach kernel and Carthamus four substance decoction for alleviating blood stasis, Chinese hawthorn fruit for removing food accumulation, gold theragran for lowering the blood lipid level, and red yeast rice for promoting circulation, dissolving stasis, and lowering blood lipid. The combination of these medicines could therefore be a practical prescription for treating stroke (phlegm and blood stasis syndrome) and a promising method for the treatment of CAP.

Modern pharmacological studies have shown that total flavonoids, triterpenoid acids of Chinese hawthorn fruit, and gold theragran could stabilize plaques and lower the level of lipids. Also, based on our clinical experience, ST 36 was effective in unblocking the meridians, quickening the collaterals, dispelling wind, and resolving dampness. ST 40 was found to reduce phlegm and lower lipids. LI 4 and PC 6 could unblock the meridians and quicken the collaterals. Our study findings suggest that combining these acupuncture points could resolve phlegm, dispel stasis, and significantly reduce tangible and intangible phlegm-blood stasis syndromes, to eventually eliminate plaques, to a certain extern.

Despite the promising results observed in this study, there were some limitations worth mentioning. As a preliminary study, the sample size was relatively small, and the follow-up time was also short. Thus, to fully determine the long-term efficacy of the therapies employed in this study and to confirm the superiority of acupuncture combined with TCM and Western drugs, compared to Western drug only, larger prospective and randomized clinical trials should be performed.

In conclusion, our findings showed that acupuncture combined with drug therapy for the treatment of CI (phlegm-blood stasis syndrome) demonstrated promising efficacies in reducing CAP volume and relieving clinical symptoms, thereby making it worthy of further clinical investigation and promising potential application.

## Figures and Tables

**Figure 1:** The study flow chart.

**Table 1:** Demographic and clinical characteristics of the included cases (*N* = 60).

Variable	Control group (*n* = 30)	Treatment group (*n* = 30)	*P* value
Gender			
Male (*n* (%))	15 (50%)	15 (50%)	>0.9999
Female (*n* (%))	15 (50%)	15 (50%)	
Age (y)	54.67 ± 9.74	54.20 ± 8.54	0.8442
Hypertension history			
Present (*n* (%))	25 (83.3%)	23 (76.7%)	
Absent (*n* (%))	5 (16.7%)	7 (23.3%)	0.5267
Diabetes history			
Present (*n* (%))	8 (26.7%)	10 (33.3%)	0.5807
Absent (*n* (%))	22 (73.3%)	20 (66.7%)	
Disease course (d)	5.35 ± 3.26	5.68 ± 3.47	0.7056
Lp-PLA2	293.5 ± 17.3	287.7 ± 16.2	0.1854

**Table 2:** Comparison of IMT of CAP between the two groups (mm).

Group	Before treatment	After treatment	*P* value
Control group (*n* = 30)	1.65 ± 0.23	1.36 ± 0.12	<0.001
Treatment group (*n* = 30)	1.71 ± 0.27	1.17 ± 0.09	<0.001
*P* value	0.3580	<0.001	

**Table 3:** Comparison of Lp-PLA2 value between the two groups.

Group	Before treatment	After treatment	*P* value
Control group (*n* = 30)	293.5 ± 17.3	179.3 ± 11.6	<0.001
Treatment group (*n* = 30)	287.7 ± 16.2	135.1 ± 10.1	<0.001
*P* value	0.1854	<0.001	

**Table 4:** Comparison of NIHSS between the two groups.

Group	Before treatment	After treatment	*P* value
Control group (*n* = 30)	28.20 ± 4.91	19.85 ± 3.03	<0.001
Treatment group (*n* = 30)	27.95 ± 4.12	11.05 ± 2.11^∗∗∗^	<0.001
*P* value	0.8316	<0.001	

## Data Availability

The data that support the findings of this study are available from the corresponding author upon reasonable request.

## Abbreviations

CAP: Carotid atherosclerotic plaque
TCM: Traditional Chinese medicine
CI: Cerebral infarction
Lp-PLA2: Lipoprotein-associated phospholipase A2
IMT: Intima-media thickness
NIHSS: National Institutes of Health Stroke Scale
ECG: Electrocardiogram
SD: Standard deviation.
